# A Review: Mechanism of *Phyllanthus urinaria* in Cancers—NF-*κ*B, P13K/AKT, and MAPKs Signaling Activation

**DOI:** 10.1155/2021/4514342

**Published:** 2021-08-26

**Authors:** Roland Osei. Saahene, Elvis Agbo, Precious Barnes, Ewura Seidu Yahaya, Benjamin Amoani, Samuel Victor Nuvor, Perditer Okyere

**Affiliations:** ^1^Department of Microbiology and Immunology, School of Medical Sciences, College of Health and Allied Sciences, University of Cape Coast, Cape Coast, Ghana; ^2^Department of Human Anatomy, Histology and Embryology, College of Medicine, Jinggangshan University, Ji'an City, Jiangxi Province, China; ^3^Department of Physician Assistant Studies, School of Allied Health Sciences, College of Health and Allied Sciences, University of Cape Coast, Cape Coast, Ghana; ^4^Department of Pharmacology, School of Medical Sciences, College of Health and Allied Sciences, University of Cape Coast, Cape Coast, Ghana; ^5^Department of Biomedical Sciences, School of Allied Health Sciences, College of Health and Allied Sciences, University of Cape Coast, Cape Coast, Ghana; ^6^Department of Medicine, School of Medicine and Dentistry, Kwame Nkrumah University of Science and Technology, Kumasi, Ghana

## Abstract

*Phyllanthus urinaria* has been characterized for its several biological and medicinal effects such as antiviral, antibacterial, anti-inflammatory, anticancer, and immunoregulation. In recent years, *Phyllanthus urinaria* has demonstrated potential to modulate the activation of critical pathways such as NF-*κ*B, P13K/AKT, and ERK/JNK/P38/MAPKs associated with cell growth, proliferation, metastasis, and apoptotic cell death. To date, there is much evidence indicating that modulation of cellular signaling pathways is a promising approach to consider in drug development and discovery. Thus, therapies that can regulate cancer-related pathways are longed-for in anticancer drug discovery. This review's focus is to provide comprehensive knowledge on the anticancer mechanisms of *Phyllanthus urinaria* through the regulation of NF-*κ*B, P13K/AKT, and ERK/JNK/P38/MAPKs signaling pathways. Thus, the review summarizes both in vitro and in vivo effects of *Phyllanthus urinaria* extracts or bioactive constituents with emphasis on tumor cell apoptosis. The literature information was obtained from publications on Google Scholar, PubMed, Web of Science, and EBSCOhost. The key words used in the search were “*Phyllanthus”* or “*Phyllanthus urinaria”* and cancer. *P. urinaria* inhibits cancer cell proliferation via inhibition of NF-*κ*B, P13K/AKT, and MAPKs (ERK, JNK, P38) pathways to induce apoptosis and prevents angiogenesis. It is expected that understanding these fundamental mechanisms may help stimulate additional research to exploit *Phyllanthus urinaria* and other natural products for the development of novel anticancer therapies in the future.

## 1. Introduction

*Phyllanthus urinaria* (Euphorbiaceae) is a traditional pharmaceutical plant that has been characterized for its several biological and medicinal effects such as antiviral, antibacterial, anti-inflammatory, and immunoregulation [1–4]. In recent years, *P. urinaria* has demonstrated to possess anticancer properties on melanoma, osteosarcoma, lung cancer, breast cancer, and prostate cancer cells [5–9]. The plant has been shown to significantly inhibit the proliferation of tumor cells via induction of apoptosis by modulating various cell signaling pathways [10, 11]. The modulation of signal transduction pathways by chemical compounds is critically important and has attained much attention among researchers. Therefore, the potential of several natural products to regulate cell signaling pathways involved in the proliferation and development of cancers has been demonstrated. To date, there is much evidence that indicates that modulation of cellular signaling transduction pathways is a promising approach to consider in drug development and discovery. This review provides comprehensive knowledge on the anticancer mechanisms of *P. urinaria* through regulation of critical pathways such as nuclear factor-kappa B (NF-*κ*B), protein kinase B (PI3K/AKT), and mitogen-activated protein kinases MAPKs (ERK/JNK/P38) with emphasis on tumor cell apoptosis.

## 2. Methodology

The literature information was obtained from publications on Google Scholar, PubMed, Web of Science, and EBSCOhost. The key words used in the search were “*Phyllanthus”* or “*Phyllanthus urinaria”* and cancer. All potential full-texts of eligible articles and research papers with title/abstract were included, and no language restrictions applied. Additional articles were obtained by tracking citations from the selected publications or directly accessing the journals' websites.

### 2.1. Apoptosis and Cancer

Apoptosis is gene-controlled programmed cell death by which multicellular organisms get rid of unwanted cells that threaten their survival, and by so doing intracellular homeostasis is maintained. Tumorigenesis, a multistep complex process that leads to malignant transformation of normal cells due to genetic alterations, is characterized by physiologic imbalance between proliferation and apoptosis. The loss of apoptosis can result in the growth of additional vasculature to provide nourishment to sustain continuous tumor growth. Apoptosis is identified by distinct morphological and biochemical hallmarks. Biochemically, it is characterized by mitochondrial release of specific mediators into the cytoplasm, stimulation of caspase mechanisms, and changes in membrane uniformity. The morphological hallmarks of apoptosis include chromatin degradation and condensation, membrane blebbing, and cell shrinkage.

Apoptosis in mammals is broadly categorized into (i) extrinsic pathway, which is initiated by the tumor necrosis factor superfamily receptors, and (ii) intrinsic pathway, which is activated by damaged DNA, and they correlate with external and internal signaling, respectively. However, the apoptotic process is highly regulated by caspases and distinct protein-protein interaction, which cooperate to activate each other in a proteolytic cascade. Apoptotic signaling activation of the caspases results in the cleavage of cellular components used for normal cell function. The apoptotic cells are then ultimately broken into apoptotic bodies, which are subsequently cleared by phagocytes via phagocytosis to prevent inflammatory response. Cancer prevention is one of the principal roles of apoptosis [12]. Deficiencies in the programmed cell death machinery of cells characterize formation of tumors and are pertinent for malignant alteration, tumor development and advancement, angiogenesis, and metastasis [13, 14]. Thus, survival and growth of most cancer cells are due to their hallmark of acquired resistance to induction of apoptosis. Dysregulation of cellular machinery involved in recognizing important extracellular and intracellular stimuli as well as signaling pathways responsible for apoptosis enable cancer cells to evade apoptosis and survive to increase their invasiveness [15]. The suppression of caspase function leads to overexpression of Bcl-2 antiapoptotic protein and underexpression of Bax and or Bak proapoptotic proteins, which affect apoptotic pathways and promote cancer cell formation [12].

### 2.2. Apoptosis and Signaling Pathways

Scientific evidence supporting apoptosis in various pathological and physiological models has provided remarkable knowledge for understanding the key functions of apoptosis in the development of cancers in humans. Activation of mechanisms regulating apoptosis can result in increased accumulation of cells or decreased cell removal.

The goal of cancer therapies is to protect normal cells without causing much damage and promote apoptosis of cancer cells. Existing cancer therapies act by direct toxicity and induction of apoptosis; hence, resistance to apoptosis may in part explain why some cancer therapeutics fail. Novel treatment approaches designed to exploit our knowledge of apoptotic mechanisms via signal transduction pathways may provide a unique therapeutic advantage for the treatment of various cancers in the future. Apoptosis can be activated and inhibited by a variety of stimuli and factors. Phenotypic features of ER-negative breast cancer occur due to unsuitable NF-kappa B signal expression and function, activating abnormal cell proliferation and inhibition of apoptosis [16]. Apoptotic signals that cause an imbalance of either declined cell death or increased cell proliferation and survival can result in cancer. The induction of continuous cell proliferation via NF-*κ*B, P13K/AKT, and MAPKs (/ERK/JNK/P38) signaling inhibits apoptosis subject to the activation of one or more pathways associated with the cell cycle. Therefore, targeting signaling pathways involved in cell proliferation, apoptosis, and differentiation may provide novel therapeutics for the treatment of cancers.

### 2.3. *Phyllanthus urinaria* Modulates NF-*κ*B, P13K/AKT, and MAPKs Activation

Tumor growth, development, and metastasis are hallmarks of aberrant gene activation of signaling pathways that subsequently predict the future of the disease. The various stages of cancer cells may be selectively hindered by several signaling transduction pathways. Recently, several studies have investigated the underlining mechanisms of *P. urinaria* and some possible targeted pathways in the treatment of cancers as shown below (Table 1).

### 2.4. NF-*κ*B Pathway

NF-*κ*B is a family of transcription factors that play a critical role in regulating different biological activities including inflammation, cell growth, and apoptosis [24, 25]. Moreover, a growing body of evidence suggests an important link between NF-*κ*B and cancer cell proliferation, development, and inhibition of apoptosis [26–29].

NF-*κ*B transcription complex in mammals comprises 5 homologous protein subunits (RelA/p65, c-Rel, RelB, p50/NF-*κ*B1, and p52/NF-*κ*B2) kept in the cytoplasm after dimerization by I*κ*Bs. Above I*κ*B bound p50, p65 dimer is the IKK complex, comprising catalytic IKK*α* and IKK*β* and regulator IKK*γ*/NEMO protein subunits [30]. IKK complex activation in response to various stimuli phosphorylates the I*κ*Bs, which subsequently targets them for ubiquitination and degradation by the 26S proteosome [31]. The liberated NF-*κ*Bs translocate to the nucleus and begin transcriptional activities of activated target genes for cellular effects such as cell growth, proliferation, apoptosis, and inflammation. NF-*κ*B is activated by a variety of stimuli and plays a critical role as both tumor promoter and suppressor [32, 33]. However, chemotherapy-induced NF-*κ*B activation is context dependent and relates to different gene expressions [34]. Therefore, NF-*κ*B inhibitors must be tried and applied with caution over prolonged period because of probable unpleasant adverse reactions. Nevertheless, natural medicines compared with their synthetic ones are thought about to have less adverse effects due to their history of prolonged usage.

Plumbagin, a plant-derived compound, dose dependently upregulated ROS and inhibited NF-*κ*B by suppressing nuclear translocation of p65 and I*κ*Bs degradation to induce apoptosis in the inhibition of lung cancer [35]. Quercetin inactivation of NF-*κ*B and activation of AP-1/JNK pathways induce apoptosis to inhibit human hepatoma cells [36]. Ellagic acid-induced apoptotic cell death on pancreatic cancer resulted from the suppression of NF-*κ*B activity [37]. The pathology of various human diseases is associated with elevated NF-*κ*B signals; hence, there is the need for techniques to inhibit NF-*κ*B events for therapeutic interventions [38]. Gene modification or pharmacological control of NF-*κ*B1 events would provide a probable therapeutic approach for several cancers [39].

The aqueous and methanolic extracts of *P. urinaria* inhibit NF-*κ*B via downregulation of p50 and p52 intracellular signals to suppress proliferation, angiogenesis, and migration in human melanoma cancer cells [11]. Tseng et al. showed that *P. urinaria* is a probable antimetastatic therapy due to its inhibition of DNA-binding action, NF-*κ*B nuclear translocation, and AP-1 in a concentration-dependent fashion. Additionally, matrix metalloproteinase-2 (MMP-2), MMP-9, urokinase plasminogen activator, and their suppressors were downregulated [18]. Prostate cancer cells treated with *P. urinaria* suppressed p50 and p52 in the inhibition of NF-*κ*B pathway via induction of apoptosis to inhibit tumor cell proliferation [17]. Corilagin downregulates the NF-*κ*B pathway to suppress cell proliferation at G2/M phase [19]. With regard to the above, it was expected that the suppression of NF-*κ*B activity by *P. urinaria* may serve to enhance the response of tumors to anticancer therapy.

### 2.5. PI3K/AKT Pathway

Phosphatase and tensin homolog (PTEN) is a tumor suppressor that negatively regulates the PI3K/AKT pathway via its capacity to transform phosphatidylinositol 3,4,5-trisphosphate (PIP3) to phosphatidylinositol 4,5-bisphosphate (PI4,5P2) [40]. The regulation of PTEN/PI3K/AKT pathway plays an important role in normal cellular activities associated with cell growth, proliferation, motility, survival, metabolism, and apoptosis.

Protein kinase B/AKTs are a set of serine-threonine kinases, which serves as the principal node of the PI3K/AKT pathway and are usually upregulated in several human cancers. AKT has three homologous isoforms—AKT 1, AKT 2, and AKT 3—which are widespread. AKT hyperactivation in cancers is due to the alteration, functional loss, or amplification of AKT 1, AKT 2, and AKT 3 genes, PTEN/P13K, and catalytic alpha polypeptide (PIK3CA) gene [41]. Erroneous activation of P13K/AKT signals play a critical function that contributes cell growth, proliferation, and suppression of apoptosis in various human cancers [42]. It has been demonstrated that PTEN upregulation inhibits cell cycle advancement and AKT phosphorylation to promote apoptosis of cancer cells [43]. PTEN deletion or functional loss hyperactivates AKT, a key downstream P13K target to induce cell growth and survival [44–47]. Hispidulin inactivates the P13K/AKT pathway in the induction of apoptosis to exert an inhibitory effect on HepG2 cells [48]. TRIM29 modulates P13K/AKT to suppress thyroid carcinoma via induced apoptosis [49]. The induction of apoptosis through the mitochondrial pathway by oxymatrine inactivated the PI3K/AKT pathway in the suppression of human osteosarcoma cell growth [50]. Zhou et al. demonstrated in both in vivo and in vitro studies that geraniin, a bioactive compound of *P. amarus*, inhibits the proliferation of colorectal cancer through induction of apoptosis by downregulating P13K/AKT activity [51].

*P. urinaria* extract inhibited the urokinase-type plasminogen (u-PA) activator in the human osteosarcoma Saos-2 cell line via suppression of AKT and ERK pathways to prevent cell invasion and migration [20]. Also, the inhibition of the PI3K/AKT, MAPKs, and hypoxia pathways by *P. urinaria* suppressed the growth of prostate cancer cells via induced apoptosis [17]. The suppression of cancers is associated with the inhibition of P13K/AKT, which is consistent with the possibility that *P. urinaria* suppresses the P13K/AKT pathway in the inhibition of tumor growth.

### 2.6. MAPKs Signaling Pathways

The mitogen-activated protein kinases (MAPKs or MAP) are a set of related protein kinases consisting of seven subgroups with three classical types including extracellular signal-regulated kinase (ERK), c-jun N-terminal kinase (JNK), and p38 MAPK, which function in cell growth, proliferation, and apoptosis. Responses of these three classical MAPKs differ in sensitivities from different cell types and different stimuli [52]. In response to different stimuli, active Ras activates Raf (MAPK KKK), which in turn activates MAPK kinases (MKKs) for transcriptional activities to produce cellular effects. MAPKs have been implicated in the development of many cancers including breast cancer, hepatoma, colon cancer, lung cancer, and liver cancer [53–57]. Ginsenoside 20(S)-protopanaxadiol is a probable therapeutic agent due to its modulation of the EGFR-mediated MAPK pathway to suppress triple-negative breast cancer [58]. Investigation has revealed that corilagin, an active ingredient obtained from *P. niruri*, blocks TGF-*β* to inactivate AKT/ERK activity to prevent ovarian cancer cell growth [59]. Teriflunomide downregulation of MMP-9, epithelial-mesenchymal transition (EMT), and inhibition of Src/FAK was achieved through the regulation of MAPK pathway to prevent the growth of cancer cell by inducing apoptosis [60]. Therefore, MAPK suppressors are being exploited as potential anticancer chemotherapeutic agents.

*P. urinaria* exertion of antimetastatic effect on lung cancer leads to the downregulation of MMP-2, MMP-7, and MMP-9 via suppression of Raf-MEK-ERK and hypoxia signaling pathways [10]. A previous report indicates that *P. urinaria* inhibited angiogenesis, proliferation, and migration of human melanoma cell via inactivation of MAPK/ERK, MAPK/P38 and upregulation of MAPK/JNK pathways [11]. Additionally, c-myc, HIF-1*α*, and VEGF expression were significantly downregulated. *P. urinaria* prevented metastasis of breast cancer through inhibition of ERK1/2 by downregulating matrix metalloprotein 2 and 9 and hypoxia pathways [21]. Geraniin, an active component of *P. urinaria*, has been reported to modulate p38 MAPK in the induction of apoptotic cell death to prevent the growth of MCF-7 [22]. Data from the treatment of human nasopharyngeal carcinoma cells suggest that *P. urinaria* gallic acid markedly suppressed AP-1/ETS-1-mediated MMP-1 transcription and matrix invasion by inhibiting the p38 MAPK pathway [23].

### 2.7. *Phyllanthus urinaria* and Apoptosis

Several important studies have scientifically proven that *P. urinaria* induces apoptosis in the inhibition of tumors. Corilagin, a bioactive compound of *P. urinaria*, induced apoptosis via both intrinsic and extrinsic pathways by downregulating procaspase-8, procaspase-3, PARP, Bcl-2, and procaspase-9 and upregulation of caspase-8, cleaved PARP, caspase-9, and Bax modulated by reactive oxygen species production in the inhibition of breast cancer cells [61]. Huang et al. demonstrated that *P. urinaria*-induced apoptosis was characterized by DNA fragmentation, membrane blebbing, and formation of apoptotic bodies in the suppression of the viability of human cancer cells [62]. In another study, Huang et al. observed that *P. urinaria* inhibits Lewis lung carcinoma proliferation by increasing caspase-3 and downregulating Bcl-2 in the induction of tumor cell apoptosis [7]. Furthermore, *P. urinaria* administration inhibited the growth of human nasopharyngeal carcinoma cell line through induction of apoptosis and decreased telomerase events by suppressing human telomerase reverse transcriptase, human telomerase-associated protein 1, and c-myc mRNA signal [63]. A more recent study [64] showed that *P. urinaria* mediates apoptosis via activation of both intrinsic and extrinsic pathways in the suppression of human osteosarcoma 143B cells [64]. Corilagin induces apoptosis by increasing caspase-3 activity to result in decreased mitochondrial membrane potential in a dose-dependent manner to inhibit ovarian cancer cells [65]. Also, *P. urinaria* alcohol extract induced apoptosis in the suppression of stomach cancer [66]. Various fractions prepared from the plant activated caspase-3 and caspase-8 and suppressed Bcl-2 to induce apoptosis in the inhibition of cancer cells via suppression of telomerase [67]. The data therefore suggest that the induction of apoptosis is one of the anticancer mechanisms of *P. urinaria* (Table 2).

### 2.8. Antiangiogenic Activity of *Phyllanthus urinaria*

Angiogenesis, the formation of additional vasculature to provide nourishment, plays a critical function in tumor development and proliferation. It is facilitated by extracellular matrix breakdown by MMP. Proangiogenic molecules such as vascular endothelial growth factor upregulate antiapoptotic proteins to aid in the survival of new endothelial cells to promote angiogenesis. The development of angiogenic inhibitors is therefore essential in the induction of tumor cell apoptosis and inhibition of metastasis. In vivo study of *P. urinaria* in mice bearing Lewis lung carcinoma resulted in significantly decreased tumor progression with marked inhibition in tumor size. Additionally, the extract inhibited tumor neovascularization and induced apoptosis with limited cytotoxicity [68]. A previous report indicates that among four *Phyllanthus* species administered on MeWo, PC-3, and human umbilical vein endothelial cells, *P. urinaria* demonstrated the strongest antimetastatic and antiangiogenic effect in a dose-dependent fashion via reduction in matrix metalloproteinase-2 [69]. The underlying mechanism of the *P. urinaria* suppression of human osteosarcoma xenograft growth in mice was due to the induction of apoptosis characterized by increased Bax/Bcl-2 ratio and inhibition of cluster of differentiation 31 via regulation of both mitochondrial fission and fusion proteins [70]. Ellagic acid, a bioactive component of *P. urinaria*, exhibits in vivo antiangiogenic effect by inhibiting MMP-2 [71]. The methanolic extract of *P. urinaria* at 100 *μ*g/mL inhibited vessel outgrowth and tube formation at 56.7% and 35.6%, respectively [72]. The aqueous extract of the plant inhibits migration and delays progression of HBV-associated hepatocellular carcinoma [73]. Tumor progression can therefore be suppressed by the regulation of angiogenesis. These results indicate that *P. urinaria* can serve as an angiogenesis inhibitor to suppress cancers (Table 3).

### 2.9. *Phyllanthus urinaria* in Clinical Trials

Traditionally, several herbal medicines are purported to have anticancer properties, and some have been proven scientifically. *P. urinaria* is claimed to possess anticancer activity as exhibited by in vitro and very few in vivo studies. To date, the few clinical trials conducted so far were carried out in hepatitis B patients. The recent clinical trial (NCT01210989) was conducted in nonalcoholic steatohepatitis patients, where 60 patients were enrolled onto a placebo-controlled parallel-group double-blind randomized controlled trial. The results revealed decreased hepatic steatosis and ballooning grades within the *P. urinaria* group, which were of limited clinical significance. Moreover, no significant difference was associated with the alterations in fasting glucose, lipid profile, alanine aminotransferase, and aspartate aminotransferase [74]. Cirrhosis patients treated with *P. urinaria* over a period of three years revealed that, compared with their controls, the extract delayed or prevented the progression of hepatitis B virus-associated cirrhosis to hepatocellular carcinoma [75]. There is therefore the need for more rigorous and effective studies of *P. urinaria* as an anticancer agent to pave way for future clinical trials.

### 2.10. Safety Profile of *Phyllanthus urinaria*

Although numerous data abound to show the therapeutic relevance of *P. urinaria* in various forms of cancer, there is paucity of evidence in the scientific literature about its toxicity profile. Most drug candidates fail to go through the drug development process due to serious toxicity. As a result, it is crucial that toxicity assessment is conducted for all promising phytochemical compounds and/or medicinal plants like *P. urinaria*. Cell viability assay with corilagin, a compound derived from *P. urinaria*, showed that it did not induce cytotoxicity in various normal human cells up to a concentration of 100 *μ*M. Furthermore, in vivo studies indicated that the compound (300 mg/kg/day) was safe in C5BL/6 mice. [76]. The ethanolic extract of the plant was found to prevent doxorubicin-induced cardiotoxicity. [77]. In a more current study, corilagin was shown to inhibit acetaminophen-induced hepatotoxicity by downregulating the inflammatory response and by inhibiting ERK/JNK MAPK and NF-*κ*B signaling pathways [78]; whereas extracts from the plant inhibited growth of breast and lung carcinoma cells, they were observed to have lower toxicity in normal cells [8]. This was a corroboration of an earlier study that reported insignificant cytotoxicity in normal human skin and prostate cells. [9]. It can be deduced from the limited available data on the toxicity of *P. urinaria* that the plant is relatively nontoxic in both in vitro and in vivo experiments. Furthermore, it has cytoprotective potential, which could prove beneficial upon exposure to various organ and cellular toxicants.

### 2.11. Future Perspective

To improve the efficacy of phytochemicals, nano-based formulation can be considered due to their potential for the treatment of several diseases and cancers. The use of natural medicine-based nanoformulations in cancer therapy has advanced and overcome the disadvantages of the conventional cancer treatment approaches such as low specificity, high toxicity, multidrug resistance, and poor bioavailability. The nonspecificity of chemotherapy has long harmed normal cell proliferation rendering cancer patients immunocompromised with long-term adverse effects. Nanomedicines have the advantages such as high proximity, high specificity, and less adverse effects, which promote their effectiveness in improving patients' response and prolonged survival. Moreover, encapsulation of bioactive components in nanocarriers can upregulate stability, extend a compound's blood circulation time, and allow for regulated and prolonged drug release in vivo. The accumulation of natural product nano-based medicines at tumor sites permits their natural components to target the cancer cells passively or actively. In vivo and in vitro studies have been used to demonstrate the anticancer effect of several nanoencapsulated natural drug products [79, 80]. Nguyen et al. reported that green silver nanoparticles formed from leaf extracts of *Phyllanthus urinaria, Pouzolzia zeylanica,* and *Scoparia dulcis* inhibited the growth of fungi [81]. Moreover, green silver nanoparticles formed from Phyllanthus amarus have also been shown to inhibit multidrug-resistant Pseudomonas aeruginosa strains [82]. Also, silver nanoparticles from *Phyllanthus niruri* leaves have exhibited excellent antibacterial activity against several multidrug-resistant pathogens in humans [83]. Reports indicate that corilagin and its metabolites have low bioavailability [84, 85]. Recently, nanotechnology-based drug delivery systems have been very promising and can change the therapeutic front of tumor cell management. Therefore, combination of nanotechnology and natural medicines such as *Phyllanthus urinaria* and corilagin as an anticancer agent may improve therapeutic response and better the clinical outcome of patients.

## 3. Conclusion

Signaling pathways in many human cancers are erroneously activated; therefore, targeting such anomalies could be of great significance to cancer treatment. NF-*κ*B, P13K/AKT, and MAPKs pathways are mostly activated in cancers, and currently few inhibitors targeting these pathways are either available or undergoing clinical trials.

This review demonstrates that *P. urinaria* inhibits cancer cell proliferation via inhibition of NF-*κ*B, P13K/AKT, and MAPKs (ERK, JNK, P38) pathways to induction of apoptosis and prevents angiogenesis. Moreover, we observed that corilagin induces apoptosis via both the intrinsic and extrinsic pathways and ellagic acid can serve as an antiangiogenic agent. Additionally, there are limited data on in vivo administration of *P. urinaria* and no clinical trials have been conducted so far with reference to cancers. The comprehensive knowledge of *P. urinaria* on these distinct molecular targets will serve as baseline data to enhance its potential and transformation for commercial use. All in all, it is expected that understanding these fundamental mechanisms may help stimulate additional research to exploit *Phyllanthus urinaria* and other natural products for the development of probable novel anticancer therapies in the future.

## Figures and Tables

**Table 1:** Modulation of critical signaling pathways by extracts or bioactive constituents of *Phyllanthus urinaria*.

Extract/bioactive constituent	Cancer type	Study type	Mechanism	Reference
Aqueous and methanolic	Human melanoma (MeWo) cancer cell line	In vitro	Suppression of NF-*κ*B, MAPKs, Myc/Max, and hypoxia pathways	[11]
Aqueous and methanolic	Human prostate adenocarcinoma	In vitro	Induce apoptosis via downregulation of NF-*κ*B, Myc/Max, hypoxia, MAPK/ERK, and MAPK/JNK	[17]
Ethanolic	Metastatic A549 and Lewis lung carcinoma and xenograft	In vitro and in vivo	Inhibition of AP-1 and NF-*κ*B binding activity	[18]
Corilagin	Glioblastoma cells U251	In vitro	Arrest cell cycle at G2/M phase and decreased NF-*κ*B pathway	[19]
Ethanolic	Human osteosarcoma cell Saos-2	In vitro	AKT and ERK pathways inhibition	[20]
Aqueous and methanolic	Human lung (A549) cancer cell line	In vitro	Raf-MEK-ERK and hypoxia pathways suppression	[10]
Aqueous and methanolic	Breast carcinoma cells (MCF-7)	In vitro	Inhibition of ERK1/2 and hypoxia pathways	[21]
Geraniin	Breast carcinoma cells (MCF-7)	In vitro	Modulation of p38 MAPK to induce apoptosis	[22]
Gallic acid	Human nasopharyngeal carcinoma cells	In vitro	Inhibition of p38 MAPK	[23]

**Table 2:** Apoptotic effects of extracts or bioactive constituents of *Phyllanthus urinaria* in cancers.

Extract/bioactive constituent	Cancer type	Study type	Mechanism	Reference
Corilagin	Breast carcinoma cells (MCF-7), MDA-MB-231 and Xenograft	In vitro and in vivo	Downregulation of procaspase-8, procaspase-3, PARP, Bcl-2, and procaspase-9 and upregulation of caspase-8, cleaved PARP, caspase-9, and Bax	[61]
Aqueous	Human cancer cells	In vitro	DNA fragmentation, membrane blebbing, and formation of apoptotic bodies	[62]
Aqueous	Lewis lung carcinoma cell line	In vitro	Induce apoptosis via downregulation of Bcl-2 and upregulation of caspase-3	[7]
Aqueous	Human nasopharyngeal carcinoma cell line	In vitro	DNA fragmentation upregulated caspase-3 and decreased Bcl-2	[63]
Aqueous	Human osteosarcoma 143B cells	In vitro	Activation of Fas receptor/ligand expression, upregulation of Bid, tBid, and Bax, and decreased Bcl-2	[64]
Corilagin	Ovarian cancer cellSKOV3	In vitro	Upregulated caspase-3 activity and loss of mitochondrial membrane potential	[65]
Alcohol	Stomach cancer cell line	In vitro	Apoptosis of MKN28 cell	[66]
Ethylene glycol, ethyl acetate, methanol, and water	HEp-2 (alveolar epithelial carcinoma cell line), MCF-7, HeLa (cervical cancer line)	In vitro	Activate caspase-3, caspase-8, and suppress Bcl-2	[67]

**Table 3:** Antiangiogenic effects of extracts or bioactive constituents of *Phyllanthus urinaria*.

Extract/bioactive constituent	Cancer type	Study type	Mechanism	Reference
Aqueous	Mice bearing Lewis lung carcinoma cells, HUVECs	In vivo and in vitro	Suppressed neovascularization in mice	[68]
Aqueous and methanolic	MeWo and PC-3HUVECs	In vitro	Suppressed of migration, invasion, and microcapillary like-tube structure formation in HUVECs	[69]
Aqueous	Human osteosarcoma xenograft mice	In vivo	Inhibition of cluster of differentiation 31	[70]
Ellagic acid	Chorioallantoic membrane in chicken embryo	In vivo	Inhibition of MMP-2	[71]
Methanolic	Male Sprague-Dawley rats, HUVECs	In vivo and in vitro	Suppression of vascular growth and tube formation	[72]
Aqueous	Hepatocellular carcinoma	In vivo and in vitro	Inhibition of migration	[73]
